# Serum 25-hydroxyvitamin D and risk of type 2 diabetes in older adults: A dose–response meta-analysis of prospective cohort studies

**DOI:** 10.1097/MD.0000000000009517

**Published:** 2018-01-05

**Authors:** Peng Cheng, Pei Fei, Yao Zhang, Zhaoxiong Hu, Hao Gong, Weijia Xu, Yujiu Gao, Qinghong Zhang

**Affiliations:** a Department of Nephrology, Taihe Hospital, Hubei University of Medicine, Hubei; b Department of Nephrology, the First Affiliated Hospital of Chengdu Medical College, Sichuan, China.

**Keywords:** dose–response relationship, meta-analysis, Type 2 diabetes, vitamin D

## Abstract

Lower serum level of 25-hydroxyvitamin D is common in older adults and associated with several negative outcomes. However, previous studies have indicated that 25-hydroxyvitamin D is associated with risk of type 2 diabetes, but presented controversial results.

Studies in PubMed and EMBASE were searched update to June 2017 to identify and quantify the potential dose–response association between low 25-hydroxyvitamin D and risk of type 2 diabetes in older adults.

Nine eligible studies involving a total of 34,511 participants with 2863 incident cases were included in this meta-analysis. Our results showed statistically significant association between lower 25-hydroxyvitamin D and type 2 diabetes in older adults [odds ratio (OR) = 1.19, 95% confidence interval (95% CI): 1.08–1.32, *P* = .001]. In addition, we obtained the best fit at an inflection point of decrease 10 ng/mL in piecewise regression analysis; the summary relative risk of type 2 diabetes in older adults for a decrease of 10 ng/mL 25-hydroxyvitamin D was 1.06 (95% CI: 1.02–1.13, *P* < .001). Furthermore, subgroups analysis indicated that lower 25-hydroxyvitamin D was associated with a significant increment risk of type 2 diabetes in older adults in female (OR = 1.21, 95% CI: 1.04–1.40, *P* = .014) but not in male (OR = 1.11, 95% CI: 0.75–1.63, *P* = .615). Subgroup meta-analyses in study design, duration of follow-up, number of participants, and number of cases showed consistent with the primary findings.

Lower 25-hydroxyvitamin D is associated with type 2 diabetes in older adults risk increment.

## Abstract 2

Supplemental Digital Content is available in the text

## 1 Introduction

Type 2 diabetes is one of the most common in the elderly and has become a serious threat to older adults.^[1]^ More than 40% of type 2 diabetes are diagnosed in the elderly (aged >60 years), and the number of elderly people with type 2 diabetes is expected to increase significantly in the next 20 years.^[2]^ As type 2 diabetes has a variety of complications, there is no specific treatment, so early defense is particularly important. The etiology of type 2 diabetes involves both genetic and environmental factors. Therefore, understanding the impact of environmental factors on type 2 diabetes will help to prevent type 2 diabetes. Obesity, sedentary lifestyle, high blood pressure, and blood cholesterol levels are potential reversible/modifiable risk factors for type 2 diabetes, and also are common targets for the prevention of type 2 diabetes.^[3]^ However, successful treatment of these risk factors has been mixed, with minimal data in the elderly,^[4]^ which suggests that there may be other potential risk factors for treatment objectives.

Vitamin D is a fat-soluble vitamin, and the human body is mainly vitamin D_2_ and vitamin D_3_. The main function of vitamin D is to maintain the metabolism balance of human calcium and the formation of bone.^[5]^ In addition, vitamin D deficiency is closely related to abnormal immune function, cardiovascular disease, metabolic diseases, and tumors.^[5]^ Lower circulating 25-hydroxyvitamin D is a common condition in older people.^[6,7]^ Also, lower vitamin D level is a potential reversible/modifiable risk factors for type 2 diabetes in older adults.^[8]^

Previous studies have examined the correlation between vitamin D and type 2 diabetes risk.^[9–17]^ However, the result remains controversial. In addition, no study to clarify and quantitative assessed vitamin D in relation to type 2 diabetes risk in older adults. Thus, we performed this dose–response meta-analysis to clarify and quantitative assessed the correlation between vitamin D and type 2 diabetes risk in older adults.

## 2 Methods

This meta-analysis was conducted according to the Meta-analysis Of Observational Studies in Epidemiology (MOOSE) checklist.^[18]^ There are no ethical issues involved in our study for our data were based on published studies.

### 2.1 Search strategy

We included eligible studies to investigate the relationship between vitamin D and type 2 diabetes risk in older adults. PubMed and EMBASE were searched for studies that contained risk estimates for the outcomes of type 2 diabetes and were published update to June 2017, with keywords, including “vitamin D” OR “25-hydroxy vitamin D” OR “hypovitaminosis D” AND “diabetes” and “old” OR “elderly” OR “older” OR “aged.”

### 2.2 Study selection

Two independent researchers investigate information on the correlation between vitamin D and type 2 diabetes risk in older adults: outcome was type 2 diabetes; the relative risks (RRs) with 95% confidence intervals. Moreover, we precluded nonhuman studies, reviews, meta-analyses, editorials, and published letters.

### 2.3 Data extraction

Use standardized data collection tables to extract data. Each eligible article information was extracted by 2 independent researchers. We extracted the following information: first author; publication year; mean value of age; country; sex; cases and participants; the categories of vitamin D; RR or odds ratio (OR). According to the Newcastle–Ottawa scale,^[19]^ quality assessment was performed for nonrandomized studies.

### 2.4 Statistical analysis

We pooled RR estimates to measure the association between vitamin D and type 2 diabetes risk in older adults; the hazard ratios were considered equivalent to the RR.^[20]^ Due to different definitions cut-off points in the included studies for categories, we performed a RR estimates by the method recommended by Orsini et al.^[21]^ Dose of vitamin D was used the median vitamin D. If the median vitamin D category was not available, the midpoint of the upper and lower boundaries was considered the dose of each category. In addition, using restricted cubic splines to evaluate the nonlinear association between vitamin D and type 2 diabetes risk in older adults. This procedure treats vitamin D (continuous data) as an independent variable and logRR of diseases as a dependent variable, with both tails of the curve restricted to linear. A *P* value is calculated for linear or nonlinear by testing the null hypothesis that the coefficient of the second spline is equal to zero.^[22]^

We use STATA software 12.0 (STATA Corp, College Station, TX) to evaluate the relationships between vitamin D and type 2 diabetes risk in older adults by using Q test and *I*^2^ statistic to assess heterogeneity among studies. Sensitivity analysis was conducted to assess the stability of the results. Begg and Egger tests were used to assess the publication bias of each study. *P* < .05 was considered significant for all tests.

## 3 Results

### 3.1 Literature search results

Figure 1 shows literature research and selection. A total of 2406 studies from PubMed and 3054 studies from Embase were included. After exclusion of duplicates and studies that did not fulfill the inclusion criteria, 9 studies were chosen, and the data were extracted. These studies were published update to June 2017.

**Figure 1:** Flow diagram of the study selection process.

### 3.2 Study characteristics

The characteristics of the included studies of vitamin D and type 2 diabetes risk in older adults are summarized in the Tables 1 and 2. Among the selected studies, 2 studies from Germany, 4 from USA, 1 from New Zealand, 1 from Netherlands, and 1 from Italy, a total of 34,511 participants with 2863 incident cases were included in this meta-analysis.

**Table 1:** Characteristics of participants in included studies of serum 25-hydroxyvitamin D in relation to risk of type 2 diabetes in older adults.

**Table 2:** Outcomes and covariates of included studies of serum 25-hydroxyvitamin D in relation to risk of type 2 diabetes in older adults.

### 3.3 Overall meta-analysis

The results of lower vitamin D and the risk of type 2 diabetes in older adults are summarized in Table 3. The pooled results suggest that vitamin D is significantly associated with type 2 diabetes risk in older adults, which was suggested both by the lowest category versus the highest category (RR: 1.19; 95% CI, 1.08–1.32; *P* = .001) (Table 3). We found no evidence of between-study heterogeneity (*I*^2^ = 0.0%, *P* = .520) and we observed no evidence of publication bias (Egger asymmetry test, *P* = .185) (supplementary Table 2).

**Table 3:** Stratified analyses of relative risk of type 2 diabetes in older adults.

### 3.4 Dose–response meta-analyses between vitamin D and type 2 diabetes risk in older adults

Using restricted cubic spline function, the test for a nonlinear dose–response relationship was significant (likelihood ratio test, *P* < .001), suggesting curvature in the relationship; decrease of 10 ng/mL vitamin D was associated with a 6% incremental in the risk of type 2 diabetes in older adults, the summary RR of type 2 diabetes in older adults for a decrease of 10 ng/mL vitamin D was 1.06 (95% CI: 1.02–1.13, *P* < .001) (Fig. 2).

**Figure 2:** Dose–response relationship between circulating 25-hydroxyvitamin D and risk of type 2 diabetes in older adults.

### 3.5 Subgroup analyses

Subgroup analysis was performed to check the stability of the primary outcome (Table 3). Subgroups analysis indicated that lower vitamin D was associated with a significant increment risk of type 2 diabetes in older adults in female (OR = 1.21, 95% CI: 1.04–1.40, *P* = .014) but not in male (OR = 1.11, 95% CI: 0.75–1.63, *P* = .615). Subgroup meta-analyses in study design, duration of follow-up, number of participants, and number of cases were consistent with the primary findings.

### 3.6 Sensitivity analysis

To explore the heterogeneity among studies of vitamin D and the risk of type 2 diabetes in older adults, we performed sensitivity analyses. A sensitivity analysis omitting 1 study at a time and calculating the pooled RRs for the remainder of the studies showed that the results were stable in supplementary Figure 1.

### 3.7 Publication bias

Each study in this meta-analysis was performed to evaluate the publication bias by both Begg funnel plot and Egger test. *P* >.05 was considered no publication bias. The results show that no obvious evidence of publication bias was found in the associations between lower vitamin D and the risk of type 2 diabetes in older adults (supplementary Table 1). A funnel plot for publication bias assessment is illustrated in Fig. 3.

**Figure 3:** A funnel plot for the meta-analysis of circulating 25-hydroxyvitamin D and risk of type 2 diabetes in older adults.

## 4 Discussion

Vitamin D is an important vitamin, mainly from fat-rich fish, butter, cheese, and fortified milk. The body itself can produce vitamin D in the sun. However, vitamin D deficiency is a common phenomenon, especially in older adults.^[5]^ It can maintain the stability of serum calcium and phosphorus levels; when the serum calcium concentration is low, it induced parathyroid hormone secretion, and released it to the kidney and bone cells. Also, vitamin D participates in critical cell functions such as cell proliferation, apoptosis, differentiation, metastasis, and angiogenesis. Vitamin D is one of the indispensable elements of health and disease prevention. Previous studies supported higher circulating 25-hydroxyvitamin D significantly decrease risk of type 2 diabetes in older adults. However, the result remains controversial.

The current meta-analysis was based on 9 cohort studies, with 34,511 participants and 2863 cases from 5 countries. Thus, this meta-analysis provides the most up-to-date epidemiological evidence supporting that lower vitamin D may be a potential risk factor for type 2 diabetes. A dose–response analysis revealed that a per 10 ng/mL of vitamin D decrease was associated with a 6% increment of type 2 diabetes risk. It is noteworthy that none of the studies reported a significant association between lower vitamin D and type 2 diabetes after adjusting for the presence of potential confounders.

Several plausible pathways may reasonable for the relationship between vitamin D and type 2 diabetes risk in older adults. Previous studies have shown that the target gene of vitamin D is a variant peroxidase proliferation activation receptor *PPARD*, which is significantly associated with insulin sensitivity. The present study determined that PPARD mutation is associated with type 2 diabetes in Han nationality.^[23]^ Second, there is a potential relationship between vitamin D and vitamin D receptor genetic polymorphism and insulin resistance in patients with vitamin D deficiency.^[24]^ In addition, the risk of vitamin D is negatively correlated with type 2 diabetes, which may be due to the clinical medium, which is related to c-reactive protein, interleukin 6, and soluble intercellular adhesion factor 1.^[25–28]^

To our knowledge, this is the first study to identify and quantify the potential dose–response association between lower vitamin D and type 2 diabetes in older adults in a large cohort of both men and women. Although we performed this meta-analysis very carefully, however, some limitations must be considered in the current meta-analysis. We only selected literature that was written in English, which may have resulted in a language or cultural bias, and other languages should be chosen in the future.

In conclusion, our dose–response meta-analysis suggests that higher vitamin D was independently associated with deleterious lung cancer decrement. However, large sample size and more studies are warranted to validate this association.

## Supplementary Material

Supplemental Digital Content
